# Association between Cardio-Ankle Vascular Index and Masked Uncontrolled Hypertension in Hypertensive Patients: A Cross-Sectional Study

**DOI:** 10.1155/2022/3167518

**Published:** 2022-12-12

**Authors:** Ning Wang, Ying Guo, Xueting Li, Ying Dong, Qi Liu, Guohong Wang, Lirong Liang, Mingzhao Qin, Qian Liu, Jiuchang Zhong

**Affiliations:** ^1^Heart Center and Beijing Key Laboratory of Hypertension, Beijing Chao-Yang Hospital, Capital Medical University, Beijing 100020, China; ^2^Department of Geriatrics, Beijing Tongren Hospital, Capital Medical University, Beijing 100730, China; ^3^Department of Clinical Epidemiology, Beijing Institute of Respiratory Medicine and Beijing Chao-Yang Hospital, Capital Medical University, Beijing 100020, China; ^4^Department of Cardiology, Beijing Chao-Yang Hospital, Capital Medical University, Beijing 100020, China

## Abstract

Detection of masked uncontrolled hypertension (MUCH) that was defined for treated hypertensive individuals who had normal office blood pressure (BP) but elevated ambulatory BP remains largely challenging. Arterial stiffness is one of the leading risk markers for hypertension and can be clinically assessed by the cardio-ankle vascular index (CAVI). This study aimed to evaluate the association between CAVI and MUCH. A total of 155 hypertensive patients were included with their office BP levels and ambulatory BP monitoring measurements, which were divided into controlled hypertension (CH), MUCH, and sustained uncontrolled hypertension (SUCH) groups, respectively. There were 48 patients with CH, 56 patients with MUCH, and 51 patients with SUCH. Both MUCH and SUCH groups had a significantly higher CAVI than the CH group (9.05 (8.20–9.91) vs. 8.33 (7.75–9.15), *p* = 0.017, and 9.75 (8.35–10.50) vs. 8.33 (7.75–9.15), *p* = 0.002, respectively). There was no significant difference in CAVI values between the MUCH and SUCH groups. Multinomial logistic regression analysis exhibited that compared with the CH group, increased CAVI levels were positively associated with the presence of MUCH and SUCH (OR 2.046, 95% CI (1.239–3.381), *p* = 0.005; OR 2.215, 95% CI (1.310–3.747), *p* = 0.003) after adjusting for confounders. However, there was a similar trend of the CAVI in the MUCH and SUCH groups (OR 0.924, 95% CI (0.629–1.356), *p* = 0.686). In summary, our findings support, for the first time, the novel notion that CAVI as an arterial stiffness parameter is an independent risk factor for MUCH, being equally important to MUCH and SUCH. When the assessed CAVI is high in hypertensive patients with normotensive office BP levels, it is necessary to further investigate with a 24 h ambulatory BP monitoring to estimate the longstanding BP control. CAVI may be used as a noninvasive indicator to identify patients with MUCH earlier.

## 1. Introduction

High blood pressure (BP) is a modifiable but poorly controlled risk factor for cardiovascular morbidity and mortality in China and worldwide. Uncontrolled BP is associated with a higher incidence of hypertension-mediated target organ damage [1]. Masked hypertension (MH), also called masked uncontrolled hypertension (MUCH) in treated patients, can be found in approximately 15% of patients with normal office BP [2]. Notably, the risks of cardiovascular events are substantially greater in patients with MH compared with the normotensive population and are actually close to or greater than those with sustained hypertension [3–6].

Patients with MH have a normal office BP albeit an elevated out-of-office BP while monitored using 24 h ambulatory BP monitoring (ABPM) or home BP monitoring (HBPM). ABPM measurement is more closely associated with hypertension-mediated target organ damage and the risk of cardiovascular events, is more reproducible than office BP measurement, and can help identify MUCH in treated hypertensive subjects [7]. However, ABPM measurement is limited often due to time restraints and intolerances when wearing [8]. Most hypertension screening and BP control assessments use office BP measurement, which is usually normal in patients with MH or MUCH. The number of patients with MUCH has been underestimated due to the lack of ABPM used to assess BP control in seemingly well-treated patients. Greater recognition and identification of MUCH can reduce the incidence of hypertension-related complications and improve their quality of life.

Increased arterial stiffness is an independent predictor of cardiovascular complications [9, 10]. Cardio-ankle vascular index (CAVI) has been proposed as an index of arterial stiffness based on the stiffness parameter *β* [11]. CAVI is easy to measure and highly reproducible. It is influenced by chronic exposure of the arterial wall to increased BP but is essentially independent of BP at the time of measurement. Some studies have reported that CAVI is high in hypertensive patients, especially in those with uncontrolled hypertension [12–14]. However, the relationship between MUCH and CAVI is largely unclear. The aim of the present study is to explore whether a high CAVI value is associated with the presence of MUCH and to evaluate the independent effect of CAVI on MUCH in hypertensive patients.

## 2. Materials and Methods

### 2.1. Study Population and Design

This was a cross-sectional study with the recruitment of the subjects being carried out in the Department of Geriatrics ward in Beijing Tongren Hospital from June 2021 to May 2022. This work was approved by the Ethics Committee of Beijing Tongren Hospital (NO. TRECKY 2021-172).

24 h ABPM and office BP levels were examined for all patients with hypertension. The inclusion of patients was the presence of a verified diagnosis of essential hypertension and receiving antihypertensives for a year or above. The exclusion criteria were listed as follows: secondary hypertension, acute coronary syndrome, chronic heart failure, cerebrovascular disease including stroke or transient ischemic attack, peripheral arterial disease, and chronic kidney disease with a decrease in glomerular filtration rate (GFR < 45 ml/min/1.73 m^2^), ankle-brachial index ≤ 0.9, acute infectious diseases, and malignant neoplasms.

According to the 2018 European Society of Cardiology/European Society of Hypertension (ESC/ESH) Guidelines for the Management of Arterial Hypertension [2], all patients were divided into controlled hypertension (CH), MUCH, and sustained uncontrolled hypertension (SUCH) groups, respectively. CH was defined as office BP < 140/90 mmHg and the mean 24 h ABPM, daytime ABPM, and nighttime ABPM are at the normal level. MUCH was diagnosed in these patients if despite controlled office BP, the mean 24 h ABPM and/or daytime ABPM and/or nighttime ABPM remained elevated (24 h systolic BP (SBP) ≥ 130 mmHg and/or 24 h diastolic BP (DBP) ≥ 80 mmHg and/or daytime SBP ≥ 135 mmHg and/or daytime DBP ≥ 85 mmHg and/or nighttime SBP ≥ 120 mmHg and/or nighttime DBP ≥ 70 mmHg). SUCH was diagnosed with both uncontrolled office and ambulatory BP.

### 2.2. Data Collection

All participants received a standardized examination. Medical information regarding age, gender, tobacco smoking, drinking consumption, duration of hypertension, medications, history of diabetes mellitus, coronary heart disease, dyslipidemia, and atrial fibrillation were extracted from the hospital's electronic medical records database. Two authors reviewed the medical data separately.

Standard instruments were used for all measurements. Anthropometry included height, weight, and body mass index (BMI; weight (kg)/height squared (m^2^)). Biochemical values included fasting blood glucose (FBG), glycated hemoglobin (HbA1c), lipid profiles including triglycerides (TG), total cholesterol (TC), high-density lipoprotein cholesterol (HDL-C), low-density lipoprotein cholesterol, (LDL-C), lipoprotein (a) (LP (a)), uric acid (UA), creatinine, and high-sensitivity C-reactive protein (hs-CRP). Blood samples were collected from the forearm vein into vacuum tubes after an overnight fast. All blood samples were measured by an automatic biochemical analyzer (AU5821, BECKMAN, USA) in Beijing Tongren Hospital Clinical Laboratory. The estimated glomerular filtration rate (eGFR) was calculated using the Chronic Kidney Disease Epidemiology Collaboration equation [15]: eGFR = 141 × min (creatinine/*κ*, 1) *α* × max (creatinine/*κ*, 1) − 1.209 × 0.993 age × 1.018 (if female). In this equation, *κ* is 0.7 if male and 0.9 if female, *α* is −0.411 if male and −0.329 if female, and min and max mean the minimum and maximum values, respectively.

### 2.3. Office BP and 24 h ABPM Measurements

Office BP measurement was taken by trained nurses. Patients sat quietly for 10 min before measurements, and the appropriate cuff size was used with the bladder encircling at least 80% of the same arm (Omron HEM-7051, Tokyo, Japan). The patient's arm was placed on the desk at the heart level. Three readings with a 1-minute interval between measurements were performed, and the last two readings were averaged as office BP [7].

24 h ABPM measurement, belonging to out-of-office BP measurements, was performed based on the 2020 International Society of Hypertension Global Hypertension Practice Guidelines [7]. An ambulatory BP monitor (Vasomedical BIOX Ambulatory Blood Pressure Monitor) was installed over the passive arm of each patient to automatically measure and record BP. In the daytime, it was programmed to perform measurements every 20 minutes between 08 : 00 and 22 : 00. In the nighttime, it was programmed to perform measurements every 60 minutes after 22 : 00. If a record contained 70% of the programmed readings, the coverage time was greater than 20 hours, and there were at least 20 readings during the day and at least 7 readings during the night, the record was considered effective. Average BP values were usually provided for daytime, nighttime, and 24 h.

### 2.4. CAVI Measurement

CAVI was measured using a VaSera VS-1000 vascular screening system (Fukuda Denshi Co, Tokyo, Japan). The patient rested on a bed in a supine position for 10 minutes before the measurements. The CAVI examination was carried out strictly in line with the operational procedure: in a quiet environment, both ankles and brachium were secured with cuffs. Electrodes for electrocardiography were placed on both wrists, and a microphone was placed on the sternum for phonocardiography.

The CAVI value was based on the stiffness parameter calculated using the following formula: CAVI = *a*{(2*ρ*/Δ*P*) × ln (*Ps*/*Pd*) × PWV^2^} + *b*, where *ρ* is blood density, *Ps* refers to the systolic blood pressure, *Pd* refers to the diastolic blood pressure, Δ*P* = *Ps* − *Pd*, PWV is pulse wave velocity between the aortic and ankle values, and *a* and *b* are constants. The CAVI value was calculated as the average of the right and left CAVI measurements. The normal value of CAVI (low CAVI) is <9, and a CAVI ≥9 is defined as the abnormal value (high CAVI) [16].

### 2.5. Statistical Analysis

The type of distribution of quantitative variables was analyzed using the Shapiro–Wilks or Kolmogorov–Smirnov tests. Continuous variables with normal distribution or with non-normal distribution were expressed as the mean ± SD or median with interquartile ranges (25th and 75th percentiles), respectively. Among the three groups, comparisons of continuous variables with normal distribution were carried out by ANOVA. The Kruskal–Wallis test was performed to compare groups with non-normal distribution. Categorical variables were expressed as the number and percentage of cases, and between-group differences were analyzed by the chi-square test or Fisher's exact test as appropriate. The Bonferroni correction was used for all pairwise comparisons. The Spearman correlation was used to identify the relations between the CAVI and BP parameters. Multinomial logistic regression analysis was performed to determine whether CAVI was independently associated with MUCH. Three models were constructed step-by-step. A *p*-value of less than 0.05 was considered statistically significant. Statistical analysis was conducted in SPSS 27.0 (SPSS Inc., Chicago, USA). Graphs were plotted using the GraphPad Prism software version 9.0 (California, USA).

## 3. Results

### 3.1. Clinical Characteristics and Biochemical Measurements of Different BP Phenotypes

After excluding 42 participants following our exclusion criteria, a total of 155 participants comprising 48 controlled hypertensive cases, 56 patients with MUCH, and 51 patients with SUCH were included in the subsequent analysis. The average age of patients was 64 years, and 110 (71%) of the patients were male.

Table 1reveals that there were no significant differences in terms of age, BMI, smoking history, drinking history, course of hypertension, comorbidities (including diabetes mellitus, coronary heart disease, dyslipidemia, and atrial fibrillation), the use of *β* blocker, antiplatelet agents, and statins. In addition, the values of FBG, HbA1c, creatinine, eGFR, UA, LP (a), TC, and LDL-C were comparable among the groups. But patients with MUCH were more likely to be male than the patients with SUCH. At the same time, there was a higher level of TG and a lower level of HDL-C in the MUCH group than in the CH group. Patients with MUCH and SUCH had a higher rate of the use of angiotensin-converting enzyme inhibitor (ACEI) or angiotensin II receptor blocker (ARB), while most of the patients in the SUCH group used calcium channel blocker agents (CCB). Both TG and hs-CRP values were higher in the SUCH group than those in the CH group.

### 3.2. Office BP and ABPM Parameters of Different BP Phenotypes

In our study, patients in the SUCH group had the highest levels of BP parameters including office SBP, office DBP, 24 h SBP, 24 h DBP, daytime SBP, daytime DBP, nighttime SBP, and nighttime DBP among the three groups (all *p* < 0.001). Compared with the CH group, the MUCH group had higher levels of 24 h SBP, 24 h DBP, daytime SBP, daytime DBP, nighttime SBP, and nighttime DBP (all *p* < 0.05), while the levels of office BP (both office SBP and office DBP) did not differ significantly between the two groups (Table 1).

### 3.3. Correlation between CAVI and Each BP Parameter in Patients with CH, MUCH, and SUCH

Spearman correlation analysis was used to examine the correlations between the CAVI and BP parameters including office BP levels and ABPM measurement (Figures 1(a)–1(d)). The level of CAVI was positively related to 24 h SBP, daytime SBP, and nighttime SBP (all *p* < 0.001). However, there were no significant correlations between office BP, 24 h DBP, daytime DBP, nighttime DBP, and the CAVI values.

### 3.4. Comparation of the CAVI for Patients with CH, MUCH, and SUCH

Both MUCH and SUCH groups had significantly higher CAVI values than that in the CH group (9.05 (8.20–9.91) vs. 8.33 (7.75–9.15), *p*=0.017, and 9.75 (8.35–10.50) vs. 8.33 (7.75–9.15), *p*=0.002, respectively). However, there was no significant difference in CAVI values between the MUCH and SUCH groups (Figure 2(a)). Of the 48 patients with CH, 15 (31.3%) had a high CAVI. Additionally, 31 cases (55.4%) had a high CAVI in the MUCH group of 56 subjects and 30 cases (58.8%) in the SUCH group, exhibiting that the trend to the high CAVI in the MUCH group was significantly higher than that in the CH group (*χ*^2^ = 6.089, *p*=0.014). However, there was no significant difference in comparison with the SUCH group (*χ*^2^ = 0.131, *p*=0.718), as is illustrated in Figure 2(b).

### 3.5. The Association between CAVI and Different BP Phenotypes

Figure 3 demonstrates the results of the multinominal logistic regression analysis of the CAVI value for the different BP phenotypes. Univariate logistic regression analysis showed that the increase of CAVI was significantly and positively associated with the MUCH(OR 1.501, 95% CI (1.106–2.036), *p* = 0.009, Figure 3(a)). After adjustment for age, sex, duration of hypertension, smoking history, the use of ACEI/ARB and CCB, higher level of CAVI remained significantly associated with the presence of MUCH (OR 2.046, 95% CI (1.239–3.381), *p* = 0.005, Figure 3(a)). Compare with CH, increased CAVI levels were positively associated with the presence of SUCH after adjusting for confounders (OR 2.215, 95% CI (1.310–3.747), *p* = 0.003, Figure 3(b)). However, there was a similar trend of the CAVI in the MUCH and SUCH groups (OR 0.924, 95% CI (0.629–1.356), *p* = 0.686, Figure 3(c)).

## 4. Discussion

Our findings suggested that the CAVI value is positively related to ambulatory SBP profiles but not associated with office BPs and ambulatory DBPs. In patients with MUCH, there is a higher CAVI value compared with patients with CH. However, there is no significant difference in CAVI values between the MUCH and SUCH groups. After adjusting for confounders, increased CAVI levels are positively and independently associated with the presence of MUCH, although there is a similar trend of the CAVI in the MUCH and SUCH groups.

MUCH in hypertensive patients is defined as normal office BP but elevated out-of-office BP (including HBPM or ABPM), among which the risk of cardiovascular events is close to or even greater than that of SUCH. Based on the use of office BP to monitor BP control, physicians will substantially overestimate the number of patients who have well-controlled BPs, leaving many higher-risk patients at an excess risk [17]. It is of great importance for MUCH to be accurately detected so that medication can be adjusted accordingly.

The clinical characteristics of patients with MH and MUCH are poorly defined [18]. Available 24 h ABPM-based studies have identified that high-normal office BP, age, male, smoking, obesity, diabetes, proteinuria, and high cardiovascular disease risks were associated with MH [19–22]. In our present study, we identified the clinical profiles of MUCH patients as more likely to be male, low HDL-C, and high TG. Notably, we observed that the office BP in the CH and MUCH groups were similar. However, those with MUCH had significantly higher levels of 24 h SBP, 24 h DBP, daytime SBP, daytime DBP, nighttime SBP, and nighttime DBP than patients with CH, which is consistent with the recently published research [21]. The findings indicated that MUCH has a negative impact on blood vessels and results in subsequent damage to multiple organs.

Arterial stiffness is becoming increasingly important in clinical applications as an early marker of hypertension-mediated target organ damage [2]. Some studies have reported that CAVI is high in hypertensive patients, especially in those with uncontrolled hypertension [12]. However, the magnitude of the relationship between arterial stiffness and MUCH is poorly reported. Previous studies found that the BP level was associated with arterial stiffness, and showed prognostic information, based only on office BP measurements [14], or arterial stiffness was mostly measured by carotid-femoral PWV [23, 24]. One study reported that CAVI was almost linear in relation to SBP, DBP, and mean BP [14] based on the office BP. In our study, we found the CAVI value was positively related to ambulatory SBPs (including 24 h SBP, daytime SBP, and nighttime SBP) but not associated with office BPs and ambulatory DBPs (including 24 h DBP, daytime DBP, nighttime DBP) in hypertensive patients. In a recent meta-analysis, the association between SBP and the progression of arterial stiffness assessed by PWV was found, while the correlation between mean arterial pressure or DBP and PWV was weak because of limited data [25].

CAVI is regarded as an arterial stiffness parameter independent of the time of its measurement, with advantages including being noninvasive, easier to obtain, and representing a global index of both central and peripheral stiffness. It thus appears to be a suitable candidate for the routine evaluation of vascular organ damage and the estimation of cardiovascular risk, especially in hypertensive subjects [26]. 24 h ABPM is an accurate assessment of BP levels, which provides plenty of information on the systolic and diastolic day and night BP profiles and ambulatory average BP levels [27], and is of great use in the identification of MH and MUCH. Due to the limited availability of ABPM, it is necessary to look for simple and noninvasive approaches to identify MUCH early in clinical practice. In this study, we found that the CAVI value was significantly higher in the MUCH group than that in the CH group, but it was similar between the MUCH and the SUCH groups. The trend of the high CAVI in the MUCH group was also higher than that in the CH group. Furthermore, adjusting for covariables of age, sex, duration of hypertension, smoking history, and the use of ACEI/ARB and CCB, the increase of CAVI is still positively associated with the MUCH compared with the CH. Until now, it is unclear whether arterial stiffness is a cause or a consequence of hypertension or whether arterial stiffness and hypertension are mutually reinforcing [28]. Findings from our current study support the notion that CAVI, as an arterial stiffness parameter, is an independent risk factor for MUCH and it is equally important to MUCH and SUCH. We recommend that even in treated hypertensive patients with normotensive office BPs when the assessed CAVI is high, patients should have a further 24 h ABPM to estimate the longstanding BP control.

## 5. Limitations

The current study has several limitations that must be taken into account. Firstly, the recruitment of the subjects was based on hospitalized patients, which may have unpredictable selection bias. Secondly, the participants might have some activities during ABPM, which to some extent may affect the accuracy of the measurement results. Thirdly, cross-sectional studies could not evaluate the causal relationship directly. Finally, the sample size of this work was relatively small.

## 6. Conclusions

Our findings support, for the first time, the novel notion that CAVI as an arterial stiffness parameter is an independent risk factor for the presence of MUCH, and that it is equally important to MUCH and SUCH. In future clinical work, when the assessed CAVI is high and above the normal range in hypertensive patients with normotensive office BP, it is necessary to further investigate with a 24 h ABPM to estimate the BP control. In hypertensive patients with normotensive office BPs, CAVI might be a potential noninvasive measurement to help identify MUCH earlier. In the future, larger prospective cohort studies are needed to further confirm the causal relationship between CAVI and MUCH among the hypertensive population. The detection of MUCH using deep learning can be the new direction [29].

## Figures and Tables

**Figure 1:** Nonparametric Spearman correlation analysis between the CAVI value and each BP parameter including (a) office SBP and DBP, (b) 24 h SBP and DBP, (c) daytime SBP and DBP, (d) nighttime SBP and DBP. BP, blood pressure; SBP, systolic blood pressure; DBP, diabolic blood pressure; ABPM, ambulatory blood pressure monitoring; CAVI, cardio-ankle vascular index.

**Figure 2:** The difference of the CAVI among patients with CH, MUCH, and SUCH. (a) Comparison of the CAVI values among the three groups. The box-whiskers plot shows the 25th and 75th percentile range (box) and median values (transverse lines in the box). (b) Comparison of the prevalence of high CAVI and low CAVI among the three groups. CH, controlled hypertension; MUCH, masked uncontrolled hypertension; SUCH, sustained uncontrolled hypertension; CAVI, cardio-ankle vascular index.

**Figure 3:** Multinomial logistic regression of the CAVI value for different blood pressure phenotypes. (a) The odds ratios of CAVI for MUCH versus CH. (b) The odds ratios of CAVI for SUCH versus CH. (c) The odds ratios of CAVI for MUCH versus SUCH. Model 1: adjusted for age and sex. Model 2: adjusted for all factors in model 1 plus duration of hypertension and smoking. Model 3: adjusted for all factors in model 2 plus the use of ACEI/ARB and CCB. CH, controlled hypertension; MUCH, masked uncontrolled hypertension; SUCH, sustained uncontrolled hypertension; CAVI, cardio-ankle vascular index; ACEI, angiotensin-converting enzyme inhibitor; ARB, angiotensin II receptor blocker; CCB, calcium channel blocker.

**Table 1:** Clinical characteristics, biochemical measurements, and BP parameters among patients with CH, MUCH, and SUCH.

Variables	CH group (*n* = 48)	MUCH group (*n* = 56)	SUCH group (*n* = 51)	*p*-value
Age (years)	62.40 ± 10.67	64.16 ± 14.26	65.61 ± 13.62	0.473
Male, *n* (%)	31 (64.6)	47 (83.9)^**c**^	32 (62.7)	**0.027**
BMI (kg/m^2^)	25.04 (23.44–26.13)	24.53 (22.48–27.35)	24.97 (23.83–26.15)	0.363
Smoking, *n* (%)	10 (20.8)	16 (28.6)	13 (25.5)	0.662
Drinking, *n* (%)	17 (35.4)	21 (37.5)	18 (35.3)	0.885
Course of hypertension (years)	4.5 (1–15)	10 (1–20)	10 (1–20)	0.07

*Clinical history, n (%)*				
DM	21 (43.8)	33 (58.9)	29 (56.9)	0.255
CHD	7 (14.6)	15 (26.8)	12 (23.5)	0.307
Dyslipidemia	37 (77.1)	48 (85.7%)	43 (84.3)	0.473
AF	4 (8.3)	3 (5.4)	2 (3.9)	0.641

*Medications, n (%)*				
ACEI/ARB	12 (25)	30 (53.6)^**a**^	31 (60.8)^**b**^	**0.001**
*β* blocker	19 (39.6)	19 (33.9)	19 (37.3)	0.834
CCB	11 (22.9)	22 (39.3)	31 (60.8)^**b,c**^	**0.001**
Antiplatelet agents	14 (29.2)	21 (37.5)	21 (41.2)	0.446
Statin	29 (60.4)	44 (78.6)	39 (76.5)	0.085

*Biochemical measurements*				
FBG (mmol/L)	5.36 (5.0–5.8)	5.75 (5.0–6.8)	5.9 (5.2–6.9)	0.187
HbA1c (%)	5.8 (5.5–6.1)	5.95 (5.7–7.8)	6.1 (5.7–6.7)	0.073
Cr (*μ*mol/L)	72.65 ± 11.26	76.42 ± 12.79	73.28 ± 13.04	0.248
eGFR (ml/min/1.73 m^2^)	86.14 ± 15.67	81.23 ± 2.33	78.96 ± 17.03	0.101
UA (*μ*mol/L)	338.5 (268–384)	356 (315–408)	350.6 (298.0–411.3)	0.259
hs-CRP (mg/L)	0.5 (0.3–1.1)	0.8 (0.4–1.5)	0.8 (0.5–2.1)^**b**^	**0.034**
LP (a) (mg/dL)	7.0 (4.3–15.2)	5.8 (3.1–18.9)	7.7 (4.0–19.6)	0.367
TG (mmol/L)	1.17 (0.84–1.66)	1.41 (0.90–2.11)^**a**^	1.37 (0.97–1.98)^**b**^	**0.033**
TC (mmol/l)	4.13 (3.52–4.92)	4.34 (3.77–4.92)	4.12 (3.51–5.36)	0.577
LDL-C (mmol/L)	2.28 (1.78–2.80)	2.44 (1.90–3.02)	2.47 (1.77–3.17)	0.556
HDL-C (mmol/L)	1.31 (1.06–1.59)	1.10 (0.92–1.33) ^**a**^	1.15 (0.92–1.33)	**0.005**

*BP parameters (mmHg)*				
Office SBP	120 (112–128)	126 (121–133)	148 (141–155)^**b,c**^	**<0.001**
Office DBP	72.5 (66–77)	75.5 (70–81)	83 (76–89)^**b,c**^	**<0.001**
24 h SBP	113 (107–120)	127 (121–136)^**a**^	136 (129–142)^**b,c**^	**<0.001**
24 h DBP	65.5 (62–70)	76.5 (71–81)^**a**^	78 (73–83)^**b**^	**<0.001**
Daytime SBP	115 (109–122)	129.5 (123–138)^**a**^	139 (129–143)^**b,c**^	**<0.001**
Daytime DBP	66 (62–72)	78.5 (72–84)^**a**^	80 (75–88)^**b**^	**<0.001**
Nighttime SBP	108.5 (106–115)	124 (116–132)^**a**^	133 (125–140)^**b**^	**<0.001**
Nighttime DBP	63.5 (59–66)	73 (71–78)^**a**^	75 (69–81)^**b**^	**<0.001**

Data are given as mean ± SD, median (IQR), or valid percentages (*n*%). CH, controlled hypertension; MUCH, masked uncontrolled hypertension; SUCH, sustained uncontrolled hypertension; BMI, body mass index; DM, diabetes mellitus; CHD, coronary heart disease; AF, atrial fibrillation; ACEI, angiotensin-converting enzyme inhibitor; ARB, angiotensin II receptor blocker; CCB, calcium channel blocker; FBG, fasting blood glucose; HbA1c, glycated hemoglobin; Cr, creatinine; eGFR, estimated glomerular filtration rate; UA, uric acid; LP (a), lipoprotein (a); TG, triglycerides; TC, total cholesterol; LDL-C, low-density lipoprotein cholesterol; HDL-C, high-density lipoprotein cholesterol; hs-CRP, high-sensitivity C-reactive protein; BP, blood pressure; SBP, systolic blood pressure; DBP, diabolic blood pressure. ^a^MUCH versus CH, *p* < 0.05. ^b^SUCH versus CH, *p* < 0.05. ^c^MUCH versus SUCH, *p* < 0.05. The bold text means that it is statistically significant.

## Data Availability

The data that support the findings of this study are available from the corresponding author upon reasonable request. The data are not publicly available due to the information that could compromise the privacy of research participants.
